# Mediating Role of Mental Resilience between Sleep Quality and Mindfulness Level of Pregnant Women Screened by Prenatal Diagnosis

**DOI:** 10.1155/2022/7011836

**Published:** 2022-01-28

**Authors:** Jinhan Liu, Xiaoxin Yan, Liangliang Chu, Chang E. Li, Jiamin Hu, Shengqiang Zou

**Affiliations:** ^1^Department of Nursing, The Affiliated Third hospital of Zhenjiang, Jiangsu University, Jiangsu, Zhenjiang 212013, China; ^2^Department of Nursing, The First Affiliated Hospital of Shandong First Medical University, Shandong, Jinan 250014, China

## Abstract

**Objective:**

To explore the status quo of psychological resilience, mindfulness level, the sleep quality of pregnant women by Prenatal Diagnosis Screening, and the mediating effect of psychological resilience on sleep quality and mindfulness.

**Methods:**

A survey of 298 pregnant women was conducted using the psychological resilience scale, Pittsburgh sleep quality index, and the concise version of the five-factor mindfulness scale.

**Results:**

The total score of psychological resilience of pregnant women was (68.96 ± 17.27), mindfulness was (77.25 ± 12.65), the median of total sleep quality was 6, and the detection rate of sleep disorders was 31.9%. The sleep quality of pregnant women was negatively correlated with mindfulness level and psychological resilience (*p* < 0.01), and mindfulness level was positively associated with psychological resilience (*p* < 0.01). Bootstrap analysis showed that psychological resilience played an 14.1% mediating role between mindfulness and sleep quality.

**Conclusion:**

The psychological resilience of pregnant women is low, sleep quality is poor, and mindfulness is mild to moderate. Psychological resilience plays an important role in mediating between mindfulness level and sleep quality that suggests nursing staff should pay attention to and improve the psychological resilience of pregnant women screened by prenatal diagnosis to improve the mindfulness level and sleep quality of pregnant women screened by prenatal diagnosis.

## 1. Introduction

Studies at home and abroad show that about 78% to 87% of pregnant women have sleep problems during pregnancy [1, 2]. The sleep survey reported that nearly 80% of women complained about disturbed sleep during pregnancy [3]. This will increase the risk of comorbidities in pregnant women and increase the likelihood of preterm birth [4]. Clinically, pregnant women usually refuse to use psychotropic medications to treat sleep problems during pregnancy due to concerns about fetal growth and development. Mindfulness is to purposefully focus your attention entirely on the present, without attaching any judgment, perception, or awareness. Mindfulness interventions as effective drug alternative therapies have been shown to improve sleep quality [4]. Mindfulness meditation is becoming a method of mental health intervention, and theoretical concepts related to it have an effect on psychopathology [5]. Psychological resilience is a dynamic process that takes shape as a change allowing people to find balance and to evolve positively [6]. It is the product of the interaction between individuals and the environment. Improving psychological resilience help individuals reintegrate and grow in the face of difficulties [7, 8]. Psychological resilience can effectively enhance changes in the hormonal levels caused by sleep disorders. Therefore, this paper aims to understand the status of sleep quality, mindfulness level, and psychological resilience in prenatal diagnosis screening of pregnant women, and to explore the role of psychological resilience between mindfulness level and sleep quality, to provide a reference to improving the sleep quality of screening pregnant women with prenatal diagnosis.

## 2. Materials and Methods

### 2.1. Subjects

From July to September 2020, 298 pregnant women were selected from the outpatient department of obstetrics and gynecology in a tertiary hospital.

Inclusion criteria are as follows: (1) age >18 years old; (2) smooth language communication; (3) pregnant women who voluntarily participate in the study and actively cooperate; and (4) elected prenatal diagnostic screening.

Exclusion criteria are as follows: (1) pregnant women with previous mental illness; (2) low intelligence or combined with severe complications; (3) communication impairment and hearing impairment. There were no ethical conflicts in “Materials and methods.”

### 2.2. Study Tool

General data shall be designed by the researcher, including basic data of age, education level, address, living status, working status and monthly family income, pregnancy week, adverse pregnancy history, mode of pregnancy, and other relevant data.

#### 2.2.1. Five Facet Mindfulness Questionnaire-Short Form (FFMQ-SF)

The scale consists of five dimensions: observation, description, perceived action, no judgment, and no behavior, with a total of 24 items. Using a grade Likert5 score method with a total score of 24 to 120, higher scores represent higher levels of individual mindfulness [9].

#### 2.2.2. Connor Davidson Resilience Scale (CD-RISC)

Connor and Davidson developed Connor Davidson Resilience Scale (CD-RISC) in 2003 [10]. Yu and Zhang [11], a Chinese scholar, introduced and Chineseizing it. The Cronbach's alpha of the Chinese version was 0.916, and the test-retest reliability was 0.821. The scale includes three dimensions: toughness, optimism, and self-improvement, with a total of 25 items. The Likert 5-level scoring method is used, with a total score of 100 scores. The higher the score, the higher the mental Resilience.

#### 2.2.3. Pittsburgh Sleep Quality Index (PSQI)

Applied Liu and Tang's Chinese version to evaluate the sleep quality in the past month. The scale includes 19 self-assessment items and 5 other-assessment items, and the scoring items are the top 18 items in the self-assessment items. Scoring items contain 7 factors, each factor 0∼3 scores, total score range 0∼21 scores, the higher the score, the worse the sleep quality [12]. PSQI total score greater than 7 scores for poor sleep quality [13].

### 2.3. Study Method

Researchers and trained nurses distributed the questionnaire. Unified guidance is adopted. On the premise of obtaining their consent, the corresponding help was given in the questionnaire filling process, and the empty items were filled again after the inquiry. All questionnaires are returned on the spot after completion and check the completeness and quality. A total of 300 questionnaires were distributed, and 298 were effectively recovered, with an effective rate of 99.3%.

### 2.4. Statistical Method

SPSS22.0 was used for statistical analysis. Counting data were tested by the number of people, in percentage description. Measurement data are described by mean and standard deviation. Pearson correlation analysis was used to analyze the correlation between mindfulness level, psychological resilience, and sleep quality of pregnant women in prenatal diagnosis screening. The hierarchical regression analysis was used to analyze the mediating effect of psychological resilience [14], and the structural equation model was established by AMOS23.0 software. The Bootstrap method is used to further verify the result.

## 3. Results

### 3.1. General Data of Prenatal Diagnosis Screening for Pregnant Women

A total of 298 pregnant women for prenatal diagnostic screening were included in this study. Age: less than 25 years old, 1 person, 0.3%; aged 25–30, 228 person, 75.7%; aged 30–35, 67 people, 22.3%; older than 35 years, 2 people, 0.7%. Education: students in junior high school and below, 2 people, 0.7%; high school, 28 people, 9.4%; specialized schools, 96 people, 31.9%; undergraduate, 161 people, 53.5%; masters or above, 11 people, 3.7%. Address: rural areas, 44 people, 14.6%; township, 120 people, 39.9%; urban areas, 134 people, 44.5%. Living status: with parents, spouses, 70 people, 23.3%, with spouses, 211 people, 70.1%; separated from spouses, basically live alone, 17 people, 5.6%. Family monthly income: less than 5000 yuan, 22 people, 7.3%; 5000–10000 yuan, 112 people, 37.2%; 10000 to 20000 yuan, 111 people, 36.9%; 20000 to 30000 yuan, 46 people, 15.3%; more than 30000 yuan, 7 people, 2.3%. Working situation: 216 employees, 71.8%; 82 nonemployees, 27.2%. Only child: 172, 57.1%; No, 126, 41.9%. Whether the pregnancy is planned: yes, 193,64.1%; No, 105,34.9%. The mode of delivery: 234 natural births, 77.7%; 64 births by cesarean section, 21.3%. Adverse pregnancy: yes, 2, 0.7%; no, 296, 98.3%. Pregnant week: less than 13 weeks, 78 people, 25.9%; 13–28 weeks, 188 people, 62.5%; more than 28 weeks, 32 people, 10.6%. Satisfaction degree of husband-wife relationship: 250 people were satisfied, accounting for 83.1%; 48 people, general, 15.9%.

### 3.2. Prenatal Diagnosis and Screening of Pregnant Women for Psychological Resilience (Table 1)

The dimension score of the optimistic, self-improvement, as well as the tough and tensile group, was 10.59 ± 3.08, 22.46 ± 5.89, and 35.93 ± 8.94, respectively. The item average score of the optimistic, self-improvement, as well as the tough and tensile group, was 2.65 ± 0.77, 2.81 ± 0.74, and 2.76 ± 0.69, respectively.

### 3.3. Prenatal Diagnosis and Screening of Pregnant Women for Sleep Quality

The total Pittsburgh sleep quality score and the score of all dimensions of pregnant women with prenatal diagnosis is shown in Table 2, with 95 sleep disorders detected, 31.9%.

### 3.4. Prenatal Diagnosis and Screening for Maternal Mindfulness Levels (Table 3)

The dimension score of the observational dimensions, describe dimensions, known dimension of action, do not judge dimensions as well as do not judge dimensions was 15.16 ± 2.94, 16.70 ± 3.45, 13.46 ± 5.00, 13.58 ± 3.59, and 18.36 ± 3.62, respectively. The item average score of the observational dimensions, describe dimensions, known dimension of action, do not judge dimensions as well as do not judge dimensions was 3.79 ± 0.73, 3.34 ± 0.69, 2.69 ± 0.10, 2.71 ± 0.72 as well as 3.67 ± 0.72, respectively.

### 3.5. Prenatal Diagnosis and Screening of Mindfulness Level, Sleep Quality, and Psychological Resilience

The results of person correlation analysis showed that PSQI was negatively correlated with the CD-RISC score range in prenatal diagnosis screening pregnant women (*r* = − 0.426, *p* < 0.01). The PSQI was negatively associated with the FFMQ-SF score (*r* = −0.429, *p* < 0.01), and the FFMQ-SF was positively associated with the CD-RISC score (*r* = 0.373, *p* < 0.01).

### 3.6. Test of the Mediating Effect of Maternal Psychological Resilience between Sleep Quality and Mindfulness Levels

The results showed that the negative effect of mindfulness level on sleep quality decreased from −0.429 to −0.314, and the effect was still significant (*p* < 0.01), indicating that psychological resilience played a partial mediating role in the prediction of mindfulness level on sleep quality in pregnant women screened by prenatal diagnosis, as shown in Table 4. This conclusion needs to be further verified.

### 3.7. Validation of Mediating Effect Model of Psychological Resilience between Mindfulness Level and Sleep Quality in Prenatal Diagnosis Screening Pregnant Women

The structural equation model of psychological resilience, mindfulness level, and sleep quality of prenatal diagnosis screening pregnant women was established. The maximum likelihood method and AMOS23.0 software were used for mediating effect test. The path analysis is shown in Figure 1. The model absolutely fits the exponential *x*^2^/d*f* = 3.067, GFI (adaptation index) = 0.890, AGFI (adjusted fitness index) = 0.831, IFI (value is configuration) = 0.937, RMSEA (progressive square and square root) = 0.096, NFI (standard adaptation index) = 0.919, showing good data fit. As can be seen from Figure 1, the direct effect of mindfulness level on sleep quality is 0.28, and the indirect effect of psychological resilience on sleep quality is 0.141 (product of 0.47 and −0.30), accounting for 34.49% of the total effect, suggesting that psychological resilience plays a partial role between sleep quality and mindfulness level. Further interval estimation was performed using the variation correction bootstrap confidence region estimation method with a sample size selection of 5000 [15]. Under 95% CI results, the mediation of psychological resilience between sleep quality and mindfulness level was −0.146, the interval did not contain 0 (LLCI = −0.248, ULCI = −0.069), suggesting a mediation effect of psychological resilience between mindfulness level and sleep quality; the direct effect of mindfulness level on sleep quality was −0.251 and the interval did not contain 0 (LLCI = −0.435, ULCI = −0.047), indicating a significant direct effect.

## 4. Discussion

### 4.1. The Psychological Resilience Level of Pregnant Women with Prenatal Diagnosis Screening Is at a Relatively Low Level

This study showed that the psychological resilience of pregnant women in prenatal diagnosis screening was low, which was consistent with the results of Zhong et al. [16]. The score of optimism dimension was the lowest (10.59 ± 3.08), which was consistent with the study of Shang et al. [17]. The reason may be that prenatal diagnosis during pregnancy and screening of pregnant women need to face both physical and psychological pressure. As the growth of pregnancy week, pregnant women will have early pregnancy reaction, insomnia, anemia, urinary frequency, oedema, constipation, stature change, changes in hormone levels, and lack of awareness of pregnancy and childbirth. The fear of prenatal diagnosis results, resulting in negative emotions such as anxiety. Pregnant women's lack of confidence in a successful pregnancy weakened their psychological resilience. Clinical nursing staff should take positive and effective measures to establish mutual communication groups, on-demand education in pregnant schools, and one-to-one psychological counseling. While improving the nursing ability, help prenatal diagnosis screening pregnant women understand pregnancy and prenatal diagnosis-related knowledge, establish confidence in a successful pregnancy, and then improve the negative emotions of pregnant women.

### 4.2. Mindfulness Levels in Pregnant Women Screened for Prenatal Diagnosis Are Low

This study showed a prenatal diagnostic screening of pregnant women with mindfulness levels at a lower level, lower than related studies [18]. The mindfulness level of pregnant women with prenatal diagnosis is at the middle level, indicating that their self-regulation and cognitive ability need to be improved. The level of mindfulness affects individuals' cognitive patterns and negative emotions caused by sleep problems. The higher the level of mindfulness, the stronger the self-regulation ability, and the more optimistic and positive they can face difficulties [19]. The level of mindfulness can be improved through learning, and long-term mindfulness practice can give practitioners peace and tranquility [20]. Mindfulness helps sleep by detecting sleep problems and not responding to any emotions or thoughts that arise. It is also necessary to explore patterns of prenatal diagnostic screening for pregnant women to improve sleep quality through mindfulness practice. Medical staff can screen pregnant women for mindfulness levels as early as possible in prenatal diagnosis and use the hospital-community and network resources to develop appropriate interventions to bring mindfulness into life and improve sleep quality through continuous learning and self-practice in prenatal diagnosis screening pregnant women.

### 4.3. Pregnant Women Have Poor Sleep Quality

This study showed that the median sleep quality of prenatal diagnostic screening was 6 score, and the detection rate of sleep disorders was 31.9%. The results showed that the three factors namely, sleep time, sleep disorder, and daytime dysfunction scored higher, consistent with Tan et al. [21]. The causes of sleep problems in pregnant women include fear of prenatal diagnosis screening results, increased nocturia, difficulty to find a comfortable sleeping position, physical pain, and discomfort, resulting in prolonged sleep time and sleep disorders. With the development of society, more and more professional women in the workplace need to work at high intensity while taking into account, their pregnancy [2, 22, 23]. Excessive energy into work may lead to daytime dysfunction. Therefore, we should attach great importance to sleep factors during pregnancy. Clinical medical staff should thoroughly evaluate the sleep status of pregnant women in prenatal diagnosis screening. Given the relevant influencing factors, early identification and intervention should be carried out to shorten sleep latency, control sleep disorders, and reduce the incidence of daytime sleep disorders to better improve pregnant womens sleep quality in prenatal diagnosis.

### 4.4. Relevant Analysis between Sleep Quality, Mindfulness Level and Psychological Resilience

Pearson correlation analysis showed that the sleep quality of pregnant women screened by prenatal diagnosis was negatively correlated with psychological resilience. Sleep quality is negatively correlated with mindfulness and positively associated with resilience. Sleep quality was negatively correlated with mindfulness levels and positively correlated with psychological resilience. This indicates that higher the mindfulness, the better the sleep quality, and higher the psychological resilience, the higher the mindfulness. The results of hierarchical regression analysis, structural equation model, and bootstrap method show that psychological resilience is the intermediary variable of the sleep quality and mindfulness level of prenatal diagnosis and screening of pregnant women and plays a partial intermediary role, accounting for 33.49% of the total effect. This indicated that psychological resilience, as a protective factor within individuals, can enhance the positive function of the mindfulness level. In the face of pregnancy-related problems, at the same mindfulness level, pregnant women with high psychological resilience levels can take a relatively more positive attitude and response way to adapt to the current state, less affecting sleep quality. On the contrary, pregnant women with poor psychological resilience are more likely to produce destructive emotions or even psychological problems and then appear sleep disorders. Consistent with the results [24], studies have shown that psychological resilience is the protective resource for the prenatal diagnosis and screening of the sleep quality of pregnant women. For pregnant women with low mindfulness levels, the mindfulness level can be improved by improving psychological resilience and sleep quality. The limit of the study is that this study is short of scientific experiments, which made the result not so solid. Further studies are needed to confirm the opinion of these reports.

### 4.5. Summary

In conclusion, prenatal diagnostic screening for maternal psychological resilience plays a significant mediating effect between mindfulness and sleep quality. Clinical nursing staff should pay attention to improving the psychological resilience of pregnant women in prenatal diagnosis and screening, and fully explore and utilize the integration of social resources so that pregnant women in prenatal diagnosis and screening can enhance their ability to cope with state changes, maintain good mental health, and improve the mindfulness level of pregnant women, and improve sleep quality. In this study, we only selected pregnant women with prenatal diagnosis and screening in a tertiary hospital as the research object. The sampling may be biased and cannot fully represent pregnant women with prenatal diagnosis and screening. In future studies, multi-center selection samples are needed for further exploration.

## Figures and Tables

**Figure 1:** Antenatal diagnostic screening for maternal psychological resilience between mindfulness level and sleep quality.

**Table 1:** Total score of psychological resilience and scores of all dimensions of pregnant women screened after prenatal diagnosis (*n* = 298).

Project	Number of entries	Score range (scores)	Dimension score ($\bar{x}\pm s$, component)	Item average score ($\bar{x}\pm s$, component)
Optimistic	4	1∼15	10.59 ± 3.08	2.65 ± 0.77
Self-improvement	8	3∼31	22.46 ± 5.89	2.81 ± 0.74
Tough and tensile	13	6∼48	35.93 ± 8.94	2.76 ± 0.69
Total scores	25	12∼92	68.96 ± 17.27	2.76 ± 0.69

**Table 2:** Total scores of sleep quality and all dimensions of pregnant women with prenatal diagnosis (*n* = 298).

Project	Median
Sleep quality	1.00
Sleep time	1.00
Hours of sleep	0.00
Sleep efficiency	0.00
Dyssomnia	1.00
Hypnosis drugs	0.00
Day dysfunction	1.00
Total scores	6.00

**Table 3:** Total scores of mindfulness levels and all dimensions of pregnant women screened after prenatal diagnosis (*n* = 187).

Project	Number of entries	Score range (scores)	Dimension score ($\bar{x}\pm s$, component)	Item average score ($\bar{x}\pm s$, component)
Observational dimensions	4	6∼20	15.16 ± 2.94	3.79 ± 0.73
Describe dimensions	5	7∼24	16.70 ± 3.45	3.34 ± 0.69
Known dimension of action	5	5∼23	13.46 ± 5.00	2.69 ± 0.10
Do not judge dimensions	5	7∼23	13.58 ± 3.59	2.71 ± 0.72
Do not act dimension Total	5	7∼25	18.36 ± 3.62	3.67 ± 0.72
	24	50∼107	77.25 ± 12.65	3.09 ± 0.51

**Table 4:** Results of stratified regression analysis of mindfulness level, psychological resilience, and sleep quality for prenatal diagnosis (*n* = 298).

Project	Dependent variable	Argument	*β* price	*t* price	*p* price	*R* ^2^ price	*F* Price	*p* price
Step 1	Sleep quality (Y)	Mindfulness level (X)	−0.429	−8.181	0.000	0.182	66.933	0.000
Step 2	Psychological resilience (M)	Mindfulness level (X)	0.373	6.918	0.000	0.136	47.863	0.000
Step 3	Sleep quality (Y)	Mindfulness level (X)	−0.314	−5.874	0.000	0.262	53.596	0.000
		Psychological resilience (M)	−0.309	−5.746	0.000			

## Data Availability

The data used to support this study are available from the corresponding author upon request.
